# Computational Analysis of Influencing Factors and Multiple Scoring Systems of Stone Clearance Rate after Flexible Ureteroscopic Lithotripsy

**DOI:** 10.1155/2022/7879819

**Published:** 2022-09-26

**Authors:** Lei Xia, Hanqing Xuan, Yang Cao, Zhebin Du, Hai Zhong, Qi Chen

**Affiliations:** Department of Urology, Ren Ji Hospital, School of Medicine Shanghai Jiaotong University, Shanghai 200127, China

## Abstract

Our research aims at the analysis of various stone scoring systems which are referred to as STONE scoring system (SSS) in this study. GUY's scoring system and RUSS scoring system (RSS) are utilized to predict stone-free status (SFS) after surgery and problems after percutaneous nephrolithotomy (PCNL) for harder stones. The data of 68 patients with renal calculi who received FURL in Ren Ji Hospital from Jan 2020 to Mar 2021 are collected as the study subjects. There were 44 male and 24 female patients, with an average age of 55.6 ± 11.4 years. Reliability analysis of related influencing factors (IF) of stone clearance rate (SCR) and multiple scoring systems after flexible ureteroscopic lithotripsy (FURL) was performed. Relevant factors with statistical significance for postoperative SCR were selected for logistic regression analysis (RA). According to the SSS score, GSS classification, and RUSS score, the SCR after FURL was statistically analyzed. The results showed that the *P* values corresponding to stone position (lower caliceal), cumulative stone diameter (CSD), urinary tract infection, and external physical vibration lithecbole (EPVL) were less than 0.05. The area under the ROC curve of RUSS score, SSS score, and GSS grading was 0.932, 0.841, and 0.533, respectively. The main IF of SCR after FURL were stone location (lower caliceal), CSD, urinary tract infection, and EPVL. The RUSS score system was the best in the evaluation of SCR after FURL. In the previous research, the score systems such as CROES (CRS), SSS, S-ReS, C, and GSS for the prediction of SFS were compared. In our analysis, we have compared the RUSS scoring system which has proven to be giving better results as compared to SSS and GSS. We also performed the regression analysis and found that the stone location shows the strongest correlation of all the other factors for stone clearing rate.

## 1. Introduction

Urinary calculi are urinary system disease that is commonly found. The clinical study data show that the incidence percentage is between 1% and 5% [1]. According to epidemiological surveys, the disease has shown a significant upward trend in China and even worldwide in the past decade [2]. Generally speaking, urinary calculi have become a nonnegligible disease threatening human health. In recent years, the detection rate of urinary calculi has been increasing, and a variety of treatment methods have gradually emerged. However, according to the location and size of stones, the general renal calculi require surgical treatment [3]. At present, the common surgical methods in clinical practice include extracorporeal shock wave lithotripsy (ESWL), percutaneous nephrolithotomy (PCNL), and flexible ureteroscopic lithotripsy (FURL) [4]. PCNL is the medical procedure to remove the calculi. In this medical procedure, a tube is inserted into the kidney through the bladder. The kidney stones are broken. Drainage tubes are used to remove the stones. PSNL is used if the stone is too hard to break. The SFR for PCNL varies in between 85 and 93%. Some of the disadvantages include bleeding, injury to pleura, injury to surrounding organs, and infection.

ESWL is generally used when the kidney stone measures from 2 to 2.5 cms. The procedure uses high-intensity acoustic waves. It is an out-patient procedure. ESWL treatment has a stone removal rate that ranges from 50% to 75%. PSNL shows 85 and 93% SCR. Lower the SCR, lower the success rate of the medical procedure. Although ESWL has high safety, the stone clearance effect is not good [5]. FURL has numerous advantages such as being minimally invasive, flexible, and repeatable, so it has been gradually widely used in the treatment of upper urinary calculi in recent years [6].

Flexible ureteroscope can retrogradely enter the urinary tract through the natural orifice and can visually and clearly observe the lesions in the urinary tract through the visual system and lithotripsy system [7]. This method has high reproducibility during treatment, so the method also has a better therapeutic effect on special populations such as patients with renal calyceal calculi, people with bleeding tendency, people with excessive obesity, people with renal anatomical malformations, and pregnant women [8, 9]. Although FURL has many advantages, it is affected by many factors, so FURL has a large difference for SCR. It is found that the factors affecting the SCR can be summarized as follows: (1) stone: such as stone diameter and location; (2) patient: such as patient weight, whether there is hydronephrosis before treatment; (3) surgeon: the difference in the proficiency of the surgeon will lead to the difference in SCR, and the same surgeon performing stone clearance surgery at different times will also lead to the difference in SCR [10–12]. At present, most of the relevant domestic studies focus on the safety and efficacy of surgery, and there are few studies on the IF of SCR.

Clinically, surgical treatment needs a simple, effective, and accurate method to assess the postoperative SCR in order to select the best treatment. Therefore, how to predict postoperative SCR accurately and effectively has always been the focus of clinical research. At present, several clinically recognized scoring systems are as follows: (1) GSS stone grading is a relatively simple scoring system, which can accurately and objectively reflect the SCR, but it does not explain some details; for example, it does not distinguish multiple stones in different calyces and the same calyx and does not include spinal malformations. However, these patients are at high risk of renal calculi and should be included; (2) RUSS stone scoring system. Relevant clinical studies have shown that this method is suitable for all patients with FURL renal calculi; (3) SSS renal calculi scoring system. Existing studies show that this scoring system can efficiently predict the SCR of nephroscopic lithotripsy [13]. Each scoring system has its advantages and disadvantages. At present, the relevant studies mostly focus on the clinical application of each scoring system, and there are few reports on the comparative study of multiple scoring systems. In [14], the authors study predictive scores for SFR after flexible ureterorenoscopy (FURS). All four scores (SSS score, RUSS, ReSC, and Ito's nomogram) could predict SFR after FURS. In [15], the researchers assess the effect of pelvicalyceal anatomy on stone clearance in the cases with remnant fragments after flexible ureteroscopy. In [16], the authors compare the scoring systems—nephrolithometry, GSS, SSS, and CRS nomogram. They have developed a risk group stratification after assessing the accuracy in prediction for SFR and other variables concerned after surgical operation. In [17], the authors compare the different scoring systems. The pros and cons are elaborated on using different scoring systems. In [18], the authors analyze the anatomical and radiological on stone clearance. They find no statistical significance in BMI, size of the stone, and lower calyx on SCR post-ESWL.

Patients suffering from calculi who underwent FURL in Ren Ji Hospital were selected as the study subjects. The relevant clinical information of the patients was retrospectively studied, and the IF of SCR were analyzed using logistics univariate and multivariate screening. The SCR after FURL was also statistically analyzed according to the SSS score, GSS grading, and RUSS score, to analyze the reliability of different scoring methods. This will provide the basis for the diagnosis and treatment of related diseases.

Major highlights of the paper are as follows:

- Analysis of various methods for predictive scores for SFR
- Comparing the predictive scores of the RUSS scoring system, SSS, and GSS
- Identification of the correlation between different factors influencing SCR

## 2. Methodology and Materials

### 2.1. Study Samples

A total of 68 patients with renal calculi who received FURL from Jan-2020 to Mar-2021, in Ren Ji Hospital, were selected for the study purpose. There were 44 male patients and 24 female, with a mean age of 55.6 ± 11.4 years. Inclusion criteria were as follows: the patients' clinical data were complete, and the whole process was treated in Ren Ji Hospital, and primary lithotripsy was successful. Single surgeon has handled all the treatments. Surgeon is having more than 2 years of experience in flexible ureteroscopic surgery. Exclusion criteria were as follows: patients with preoperative severe renal insufficiency; patients with severe hydronephrosis; patients who underwent two or more flexible ureteroscopic surgeries; patients with sponge kidney and renal calculi; patients with ureteral stricture. The patients were split into stone clearance group (43 cases) and residual stone group (25 cases).

SCR is the ratio of the number of patients from whom the stone was removed completely to the total patients who received the treatment.

Patient signed an informed consent form, and the experiment met medical ethics requirements.

### 2.2. Surgical Methods

The patients suffering from urinary tract infection (UTI) were given sensitive antibiotics before the operation, and the operation was performed after the control of urinary tract infection. All patients were given prophylactic antibiotics 0.5–2 hours before the operation to avoid or reduce serious complications such as urosepsis.

After general anesthesia, the lithotomy position was taken, and Wolf F8/9.8 rigid ureteroscope was put in through the urethra, upward along the ureteral orifice of the affected side until the pelvis or upper ureter, and 0.035 mm nickel-titanium wire was inserted. The F12/14 flexible ureteroscope (High Quality Urology Single-Use Flexible Video Ureteroscope Digital Disposable Urethroscope, Guangzhou Lety Medical, Ltd.) sheath was introduced with the guide wire inserted into the below UPJ or ureteral calculi, the Olympus flexible ureteroscope (URF-V, F8.5-9.9) was inserted along the sheath, and the holmium laser fiber was introduced. The fiber diameter was 200 *μ*m, and the crushing of stones energy was set to (0.6–1.2) J × (16–20) Hz, and the maximum diameter of stones needed to be crushed <2 mm. At the end of the operation, each calyx of the kidney was examined again to ensure that no large stones remained. F5 ureteral stent was put in with the guide wire, and the catheter was indwelled. KUB was reexamined on the first day after FURL to evaluate the crushing of stones and the position of the ureteral stent and to guide the patient's body position according to the distribution of stones. Postoperative expulsion was carried out by referring to the method of Xu Changbao et al. on external physical vibration lithecbole (EPVL).

### 2.3. Measurement Method

There are different CT-based measurement methods to calculate stone volume. CT-based 3D-reconstructed algorithm, threshold-based methods, noncontrast helical computed tomography, and manual stone size measurements are some of the methods. [14–16].

Slice computed tomography scanner medical CT scan machine was used to scan the images.

The complete medical history data as well as imaging data such as laboratory tests and CT of each patient were used as evaluation objects. Indicators of patient and stone characteristics as independent variables were collected, and the SCR in one-stage surgery was also calculated. The relevant variables were measured according to RUSS, SSS, and GSS. The average CT value of the stone was measured according to the three areas of the maximum cross section of the stone at three levels by CT scanning, and the CT values (HU) of the core, edge, and the position between the two were recorded, respectively. The average CT value of each stone was calculated (staghorn stones could be measured by this method). The average of multiple stones was calculated. IPA is the minimum angle between the long axis of the lower calyx and the long axis of the ureteropelvic.

Stone size grading: the stones were grouped according to their maximum diameter in the CT cross section, which were divided into diameter less than 1 cm group, diameter 1-2 cm group, and diameter more than 2 cm group. All measurement data were recorded after consensus by the 2 observers.

### 2.4. Scoring Systems

GSS stone grading criteria: it was put forward by Thomas et al. in 2011 depending on the structure and stones distribution of renal pelvis and calyces. The GSS was developed after analyzing the published data review and expert opinion. Iterative testing was done. It predicts the post-PCNL SFR with great accuracy. It shows reproducibility and is easy to use. GSS score is found to be significant in predicting the SFR (*P*=0.01) independently [17]. The method is divided into four levels, and the detailed grading standards and contents are shown in Figure 1.

RUSS was first presented by Resorlu et al. in 2012. The SCR after FURL can be predicted according to the score. The high score signifies low SCR. The detailed scoring criteria are given in Figure 2.

SSS for renal calculi: the scoring system includes five items, and the postoperative SCR of PCNL can be predicted based on the score. The detailed scoring criteria are shown in Table 1.

### 2.5. Statistical Method

SPSS 22.0 is utilized in this medical research study for analysis. The data were expressed as mean ± standard deviation ($\bar{x}\pm s$), and for comparison among the groups, *t*-test was used. Variance analysis was adopted for comparison within the group; *χ*^2^ was used for counting data; *P* < 0.05 shows the difference that is statistically significant. The single factor analysis was carried out using univariate regression analysis. In univariate linear regression, we identify the correlation between single independent variable and one dependent variable. The multifactor analysis was carried out using multivariate RA. In this method, we identify the correlation between single dependent variable and multiple independent variables.

## 3. Results

### 3.1. Univariate Regression Analysis Results

We examined the CT scan reports of patients with renal calculi who received FURL from Jan-2020 to Mar-2021, in Ren Ji Hospital, were selected for the study purpose. Male patients were 44 in number, and female patients were 24 in number. Average age is 55.6 ± 11.4 years.

The univariate analysis is carried out for the IF of the stone clearing rate for the stone clearing group. The IF of the stone clearing rate were analyzed by univariate analysis, and the results were shown in Figure 3. *P* values corresponding to the location of stones, the cumulative stone diameter (CSD), urinary tract infection, EPVL, hydronephrosis, and other factors are all less than 0.05 indicating that these variables are statistically significant in the univariate RA of the IF of SCR.

The following Table 2 shows the results of univariate RA on IF of SCR.

The following Figure 3 shows the results of univariate RA on IF of SCR.

### 3.2. Results of Multivariate Regression Analysis

The IF of the stone clearing rate were analyzed by multiple factors.  Figure 4 indicates that the *P* values corresponding to stone position (lower calyx), stone diameter, urinary tract infection, and EPVL are less than 0.05, with statistical significance, which were finally included in the model. It can be concluded that the location of stones (lower calyx), the maximum diameter of stones (20–30 mm), urinary tract infection, and EPVL are the main factors affecting the SCR after FURL, and the correlation with the location of stones is the strongest.

The following Table 3 shows the multivariate RA results of IF of SCR.

The following Figure 4 shows the multivariate RA results of IF of SCR.

### 3.3. Comparison of SCR of RUSS Stone Scoring System

SCR comparison results of the RUSS stone scoring system are shown in Figure 5. The proportions of patients with RUSS scores of 0, 1, 2, 3, 4, and 5 in the stone clearance group were 55%, 36%, 36%, 1.8%, 1.8%, and 1.8%, respectively; the proportion of patients with RUSS scores of 0, 1, 2, 3, 4, and 5 in the residual stone group was 12%, 24%, 27%, 21%, 9%, and 6%, respectively. The score of RUSS in the stone clearance group was 0.57 ± 0.44, and that in the residual stone group was 2.11 ± 1.62.

Comparison of SCR of the RUSS stone scoring system is shown in Figure 5.

### 3.4. Comparison of SCR of STONE

SCR comparison results of SSS were shown in Table 2. SSS stone score in the stone clearance group was 4.33 ± 1.13, the SSS stone score in the stone residual group was 8.26 ± 2.01, and the value of P indicates a statistically significant difference between the two groups.  Table 4 shows the comparison of SCR of SSS.

### 3.5. GSS Stone-Clearance Rate Comparison Results

SCR comparison results of GSS were given in Figure 6. The proportion of patients with GSS grade One, Two, Three, and Four in the stone clearance group was 11%, 45%, 62%, and 0%, respectively; the proportion of patients with GSS grade One, Two, Three, and Four in the stone residual group was 3%, 30%, 64%, and 3%, respectively. Comparison results of GSS are shown in Figure 6.

### 3.6. ROC Curve Analysis of Each Scoring System for FURL SCR

The ROC curve analysis results of each scoring system for FURL SCR are shown in Figure 7. The ROC curve of each scoring system was 0.932, 0.841, and 0.533, respectively, and the order was RUSS > SSS > GSS. The performance of RUSS scoring system was the best, followed by SSS and GSS. ROC curve analysis of FURL SCR by each scoring system is shown in Figure 7.

## 4. Discussion

Urinary calculi are one of the general ailments of the urinary system, and the incidence of this disease in China ranges from 5% to 10%, which shows an increasing trend year by year [18]. This disease is also found amongst the children now a days.

New treatments and corresponding grading systems have also been developed. At present, the main treatment methods for the urinary system include ESWL, PCNL, and FURL. URL is currently widely used in clinical practice. FURL is widely adopted due to its characteristics of less trauma, high efficiency, and wide indications has become the treatment of option for renal calculi of 1-2 cm in diameter and is considered to be the best alternative for patients who cannot undergo PCNL. We can gauge the effectiveness of these treatments using well-known scoring methods. These methods are as follows.

1. SSS: It is simple to assess and has a good predictive value, but it does not contain abnormal renal anatomy or spinal deformity and other factors that may affect the therapeutic effect of FURL, and its predictive ability has also to be validated with a prospective, multicenter study
2. GSS grading: GSS is mainly graded according to the pelvicalyceal structure and stone distribution. For FURL, abnormal renal anatomy and different stone distribution will also affect the postoperative SCR of FURL. However, due to different positions, the surgical access channel adopted is inconsistent. GSS grading does not consider the factors such as stone size grading and stone cross-sectional area, which may be the reason for its poor effect in predicting the postoperative SCR of FURL
3. RUSS score: The RUSS scoring system is simple and practical, but its indicators do not contain other indicators that may affect the SCR such as stone hardness and the degree of hydronephrosis
4. CRS: The CRS nomogram can predict the renal stone complexity with great accuracy. Postoperative efficacy can be predicted accurately with CRS nephrolithometry
5. S-ReSC: It was developed to predict the SFR after PCNL. It also describes the complexity of renal stones [17, 18].

In the previous researches, in order to compare the scoring, the score systems such as CRS, SSS, S-ReSC, and GSS for the prediction of SFS were compared. In our analysis, we have used the RUSS scoring system which has proven to be giving better results as compared to SSS and GSS. We also performed the RA and found that the stone location shows the strongest correlation of all other factors.

## 5. Conclusion

After the analysis, the results suggest that the factors such as location of stones (lower calyx), the CSD (20–30 mm), urinary tract infection, and EPVL are the main factors affecting the SCR after FURL. The stone location is found to have the strongest correlation of all. The RUSS scoring system has proven out to be the most accurate one for the evaluation of SCR after FURL, followed by the SSS and the GSS. Our current research compares the reliability of several existing scoring systems. In our future work, we will come up with the method for improving the existing scoring system. In the future, we will consider a bigger sample size for the analysis. We also will categorize the patients in different age groups, as kidney stone is being found in the younger population as well now a day.

## Figures and Tables

**Figure 1:** GSS stone grading.

**Figure 2:** RUSS stone scoring system.

**Figure 3:** Results of univariate RA on IF of SCR. Note: CSD: cumulative stone diameter; EPVL: external physical vibration lithecbole.

**Figure 4:** Multivariate RA results of IF of SCR.

**Figure 5:** Comparison of SCR of RUSS stone scoring system. Note: (a) proportion of patients; (b) score results; compared with the stone clearance group, ^*∗*^*P* < 0.05.“*∗*” in “^*∗*^*P*” indicates that there is a significant difference between the two.

**Figure 6:** Comparison results of SCR of GSS.

**Figure 7:** ROC curve analysis of FURL SCR by each scoring system. Note: (a) ROC curve; (b) area under the curve; compared with RUSS, ^*∗*^*P* < 0.05.

**Table 1:** SSS for renal calculi.

*S*: stone size, the length × width of the largest cross-sectional area of stone in CT plain scan = cross-sectional area (mm^2^)	1 points 0∼399
	2 points: 400∼799
	3 points: 800∼1599
	4 points: ≥1600

*T*: tract length, the distance measured from the center of stone to the skin on the cross section of CT (horizontal line, 45° line, and vertical line).	1 point: ≤100 mm
	2 points: >100 mm

*O*: obstruction, degree of hydronephrosis	1 point: no obstruction or mild hydronephrosis
	2 points: moderate or severe hydronephrosis

*N*: number of involved calices	1 point: 1 renal caliceal involvement
	2 points: 2–3 renal calices involvement
	3 points: complete staghorn calculi

*E*: essence or stone density	1 point: ≤950HU
	2 points: >950HU

**Table 2:** Results of univariate RA on IF of SCR.

	*B*	Wald	Sig▪	Exp (*B*)
Gender	−0.101	0.215	0.541	0.981
Age	−0.241	0.293	0.536	0.785
BMI	−0.143	0.684	0.539	0.932
Serum creatinine	0.657	2.361	0.233	3.149
CSD	2.237	7.459	0.113	3.459
Stone position	1.934	27.53	0	7.532
Infection	0.925	6.303	0.048	3.392
Kidney seeper	0.603	5.882	0.0361	2.639
EPVL	2.077	20.657	0	5.447

**Table 3:** Multivariate RA results of IF of SCR.

	*B*	Wald	Sig▪	Exp (*B*)
Stone position	0	44.36	0	0
Renal pelvis	0.361	0.286	0.843	2.215
The calyx	3.114	30.27	0	20.117
CSD	1.13	5.366	0.058	3.116
EPVL	2.358	11.3	0.005	6.337
Constant	−7.73	30.56	0	0.005

**Table 4:** Comparison of SCR of SSS.

	Stone clearance group (*n* = 43)	Stone residual group (*n* = 25)	Total	*t*	*P*
SSS	4.33 ± 1.13	8.26 ± 2.01	—	−4.324	0.002

S				15.109	0.001
1	39 (90.7%)	15 (60.0%)	54 (79.4%)	**#####**	
2	2 (4.7%)	8 (32.0%)	10 (14.7%)		
3	2 (4.7%)	2 (8.0%)	4 (5.9%)		

T				0.067	0.833
1	31 (72.1%)	14 (56.0%)	45 (66.2%)	**#####**	
2	12 (27.9%)	11 (44.0%)	23 (33.8%)		

O				0.311	0.746
1	29 (67.4%)	15 (60.0%)	44 (64.7%)	**#####**	
2	14 (32.6%)	10 (40.0%)	24 (35.3%)		

N				14.513	0.002
1	31 (72.1%)	13 (52.0%)	44 (64.7%)	**#####**	
2	11 (25.6)	11 (44.0%)	22 (32.3%)		
3	1 (2.3%)	1 (4.0%)	2 (2.9%)		

E				5.538	0.041
1	34 (79.1%)	11 (44.0%)	45 (66.2%)	**#####**	
2	9 (20.9%)	14 (56.0%)	23 (33.8%)		

**#####** indicates that there is no relevant content.

## Data Availability

The data can be made available on valid request.
